The article "Screening of Hub Genes in Hepatocellular Carcinoma Based on Network Analysis and Machine Learning" was published in 2022. Journal: Comput Math Methods Med.

# Screening of Hub Genes in Hepatocellular Carcinoma Based on Network Analysis and Machine Learning

**DOI:** 10.1155/2022/7300788

**Published:** 2022-11-28

**Authors:** Yu Zhang, Yongfang Xie, Xiaorong Huang, Langlang Zhang, Kunxian Shu

**Affiliations:** School of Bioinformatics, Chongqing University of Posts and Telecommunications, 400000, China

## Abstract

Hepatocellular carcinoma (LIHC) is the fifth common cancer worldwide, and it requires effective diagnosis and treatment to prevent aggressive metastasis. The purpose of this study was to construct a machine learning-based diagnostic model for the diagnosis of liver cancer. Using weighted correlation network analysis (WGCNA), univariate analysis, and Lasso-Cox regression analysis, protein-protein interactions network analysis is used to construct gene networks from transcriptome data of hepatocellular carcinoma patients and find hub genes for machine learning. The five models, including gradient boosting, random forest, support vector machine, logistic regression, and integrated learning, were to identify a multigene prediction model of patients. Immunological assessment, TP53 gene mutation and promoter methylation level analysis, and KEGG pathway analysis were performed on these groups. Potential drug molecular targets for the corresponding hepatocellular carcinomas were obtained by molecular docking for analysis, resulting in the screening of 2 modules that may be relevant to the survival of hepatocellular carcinoma patients, and the construction of 5 diagnostic models and multiple interaction networks. The modes of action of drug-molecule interactions that may be effective against hepatocellular carcinoma core genes CCNA2, CCNB1, and CDK1 were investigated. This study is expected to provide research ideas for early diagnosis of hepatocellular carcinoma.

## 1. Introduction

Liver cancer is one of the most common cancers worldwide. The incidence of liver cancer accounts for 8.2% of total cancer cases and 4.7% of total cancer deaths. In some regions, the incidence rate is still increasing. Despite significant improvements in the diagnosis and treatment of liver cancer, the long-term prognosis remains poor, and liver cancer remains an important global clinical challenge [1, 2]. Therefore, the development of more sensitive diagnostic methods, the use of new biomarkers, and the construction of effective prognostic models are important to improve the survival time of patients.

Image-based algorithms drive the diagnosis of disease [3, 4]. HCC can be diagnosed based on imaging features alone, and the noninvasive nature and wide availability have led many HCC guidelines to recommend image-based diagnosis [5]. Several studies have shown good results in classifying liver cancer images by using a machine learning approach [6, 7]. Serum *α*-fetoprotein (AFP) has been widely used as a predictive and prognostic biomarker for HCC, but the sensitivity of AFP for detecting early stage HCC is limited [8, 9]. The construction of machine learning models by some candidate markers such as cell-free DNA (cfDNA) provides room for improvement in the diagnosis of HCC [10]. In recent years, the use of other samples for prediction has also shown good promise [11, 12]. However, the selection of these characteristics does not explain well the mechanism of hepatocarcinogenesis and prognostic therapies at the genetic level. RNA sequencing (RNA-seq) can reveal gene fusions, splice variants, mutations/insertions deletions, and differential gene expression, thus providing a more complete genetic map than DNA sequencing [13]. Some current statistical analyses of the hepatocellular carcinoma transcriptome suffer from the problem of focusing only on statistical results and detaching from the biological context. Machine learning is better able to deal with complex nonlinear relationships in the data than some conventional statistical tools; however, part of the models lacks explanatory power [14].

Weighted correlation network analysis (WGCNA) aggregates genes with similar expression patterns in the same genetic module and identifies relationships between gene modules and phenotypes to identify potential candidate biomarkers or novel therapeutic targets [15]. The competing endogenous RNA (ceRNA) hypothesis addresses a complex posttranscriptional regulatory network. When two transcripts contain the same miRNA response element (MRE), they can compete with a shared miRNA. This means that the upregulation of one transcript leads to the segregation of more copies of the shared miRNA, which reduces the expression of the other transcript and vice versa [16].

In this study, we screened genes with survival and other indicators by WGCNA and used univariate—Lasso—multiple Cox regression analysis and survival analysis and protein-protein interactions (PPI) to screen for signature genes. Training was performed using random forest, gradient boosting, support vector machine, logistic regression, and integrated learning. The gene characteristics are also explained by ceRNA network, pathway enrichment and TP53 mutations, promoter methylation, and immune cell infiltration. Our study is aimed at combining biology with statistics and machine learning to provide new insights into potential targets for hepatocellular carcinoma and to promote precision therapy for HCC.

## 2. Materials and Methods

### 2.1. Data Collection

The main procedure of our study is shown in Figure 1. The RNA-seq data associated with HCC were downloaded from TCGA. There were 424 lncRNA and mRNA samples, including 50 normal samples and 374 tumor samples. And 425 miRNA samples were also downloaded, including 50 normal samples and 375 tumor samples. The relevant clinical characterization data were downloaded through UCSC Xena (http://xena.ucsc.edu/). After screening, we retained 294 samples of the lncRNA and mRNA dataset (including 50 normal samples and 244 tumor samples). In machine learning, the training data is GSE76427 (including 52 normal samples and 115 tumor samples) from the GPL10558 platform, while the validation set GSE102079 (including 105 normal samples and 152 tumor samples) is from the GPL570 platform.

### 2.2. Data Preprocessing and Analysis of Differentially Expressed Genes

DEGs between tumors and adjacent tissues were identified using the R package “edgeR”. |log2 − fold change(FC)| > 1 and *p* < 0.05 were considered statistically significant. Cluster heat maps were generated using the pheatmap R package. Principal component analysis was performed by the factoextra package to visualize the data. Volcano map visualization of differential genes was performed using the ggplot package.

### 2.3. Construction of Coexpressed Gene Networks Based on WGCNA

WGCNA is an analysis method to identify gene coexpression networks based on topological overlap. The final input of 6,500 genes was made by descending order of the expression values of the dataset. WGCNA was then used to construct coexpression networks of differential genes. Coexpression gene networks were created with a soft threshold of minimum value of *R*2 > 0.9 to cluster genes with high correlation into the same module. Correlations between modules and clinical data were calculated to screen for modules associated with survival time and other prognosis or diagnosis of HCC. Finally, correlated mRNA and lncRNA were obtained.

### 2.4. Construction of RNA Network in Hepatocellular Carcinoma

The interactions between lncRNA and miRNA and miRNA and mRNA in the WGCNA module were predicted using ENCORI (http://starbase.sysu.edu.cn/index.php;version3.0). The predicted miRNAs intersected with the differential miRNAs in TCGA. In addition, the predicted RBPs that interact with the lncRNAs and mRNAs in the module were taken to intersect and merge. Finally, data on the interactions between these RBPs and mRNAs in different organs and cancer types were retrieved. These networks were visualized by Cytoscape (3.7.2). Finally, we obtained lncRNA-miRNA-mRNA, lncRNA-RBP-mRNA, and RBP-mRNA-tissue-disease networks.

We used the database search tool for retrieval of interacting genes/proteins (STRING) (https://www.string-db.org/) to evaluate protein-protein interactions (PPI) information and Cytoscape (3.7.2) for visualization. The R package “clusterProfiler” was used to perform Gene Ontology (GO) and Kyoto Encyclopedia of Genes and Genomes (KEGG) analyses [17]. GSEA (version 4.1.0) was used for gene set enrichment analysis (GSEA) [18], where we defined enrichment markers as FDR < 0.25, NOM *p* value <0.05, and |NES| > 1.

### 2.5. Construction and Validation

To minimize the risk of overfitting, Lasso-penalized Cox regression analysis was applied to construct the prognostic model. The Lasso algorithm was used for variable selection and shrinkage using the “glmnet” R package. Patients were divided into high-risk and low-risk groups based on the median risk score. The risk score was calculated as follows: riskscore = ∑(coefficienti × expression of signature genei). Differences in OS time between risk groups were analyzed using Kaplan-Meier (KM) survival analysis and log-rank test.

### 2.6. HCC Diagnostic Model Construction and Core Gene Screening

Training and test sets for model construction were divided from the dataset generated by combining the TCGA and GSE76427 datasets from the GPL10558 platform. To validate the stability of the model, we used the GSE102079 dataset from the GPL570 platform as the validation set. These data were normalized, and missing values were replaced using the average of the same genes. Random forest, gradient boosting, support vector machine, logistic regression, and integrated learning were used to train the models using the python package “scikit-learn” [19]. These models were validated by the 5-fold cross-validation method and the leave-one-out method.

### 2.7. Analysis of Key Genes and Immunological Characteristics

Analysis of TP53 mutation status (TP53 mutation status) and promoter methylation levels (promoter methylation) for normal data and hepatocellular carcinoma data was performed through the UALCAN website [20].

An immunization file on LIHC patients in TCGA was downloaded through the TIMER 2.0 website [21]. This file includes TIMER, CIBERSORT, quanTIseq, xCell, and MCP-counter [22–26]. Infiltration estimation of TCGA patients was performed with these 5 tools. RNA data were processed using the R package DESeq2 package [27], and the association between core genes and immunity was analyzed using the R package psych. Finally, heat map presentation was performed by pheatmap of R package.

### 2.8. Core Genes Targeting Corresponding Drug Candidates

Interaction studies of obtained hub genes with relevant drugs were performed to analyze their targeting effects, where candidate antihepatocellular carcinoma drugs were obtained from the DGIdb (http://www.dgidb.org/) database, an online tool containing information on drug-gene interactions from more than 30 libraries. These molecules were mainly from the ZINC library (https://zinc.docking.org/), while others were drawn by marvinsketch (version 21.9) [28], and the lowest energy conformation was selected. The conversion of mol2 files was performed using the open source chemistry toolbox open Babel (version 2.3.2) [29]. The 3D structures of the proteins expressed by the target genes were obtained from the RCSB PDB library (https://http://www.rcsb.org/). PyMOL (version 2.3) [30] removes hydrogen bonds and other ligands from the target protein. Autodocktools (version 1.5.6) [31] adds hydrogen atoms, binds nonpolar hydrogen atoms, calculates the charge number of the protein, and detects the docking sites. Finally, the target protein in pdbqt format is docked to the drug candidate by AutoDock Vina 1.1.2 [32] with a threshold of affinity -7.0 kcal/mol. The final 2D structure is drawn using ligplot (version 4.0) [33].

## 3. Results

### 3.1. Analysis of Data in TCGA-LIHC Samples

After the differential analysis of TCGA-LIHC samples, 3529 differential lncRNAs, including 3008 upregulated genes and 521 downregulated genes, were screened; 2183 differential mRNAs, including 4074 upregulated genes and 1109 downregulated genes, were obtained; 330 differential genes of miRNAs included 287 upregulated genes and 43 downregulated genes (Figure 2).

Next, GO and KEGG enrichment analyses were performed on the up- and downregulated differential mRNAs. We found that the expression of upregulated genes was mainly focused on the pathways with cell morphology, channels, and receptors. The downregulated differential genes, on the other hand, were mainly distributed in pathways related to metabolism and degradation (Figure 3). These changes may be related to disruption of liver function.

### 3.2. Cox Regression Analysis of Clinical Indicators

Cox regression analyses were performed on clinical data. The clinical information included fetoprotein outcome value, total bilirubin upper limit, bilirubin lower limit, bilirubin upper limit, age at initial pathologic diagnosis, sample type, gender, histological type, neoplasm histologic grade, platelet result count, platelet result lower limit, platelet result upper limit, and weight. The ROC curve and KM survival analysis combined with landmark analysis showed that the upper limit of total bilirubin could effectively distinguish between high-risk and low-risk patients with *p* = 0.0019 (Table 1, Figure 4). Methemoglobin is often used as a diagnostic indicator for HCC. Therefore, we selected age at initial pathologic diagnosis, bilirubin lower limit, bilirubin upper limit, survival time, fetoprotein outcome value, and total bilirubin upper limit as the clinical indicators associated with WGCNA.

### 3.3. WGCNA Expression Module Analysis

Initial screening using WGCNA selected *β* = 3 as the soft threshold of the network, and 21 gene coexpression modules were obtained by WGCNA (Table 2).

The correlation between modules and clinical characteristics was analyzed according to the clinical profile of UCSC Xena. Turquoise module was found to be highly correlated with survival time and survival status (*p* < 0.05). Also, the blue module was highly correlated with other clinical information (Figure 5(b)). The correlation between blue and turquoise modules was low (Figure 5(c)). And the topological overlap matrix (TOM) plot showed a strong coexpression relationship of genes in both modules (Figure 5(d)). Two coexpression modules were obtained, in which lncRNAs and mRNAs were HCC survival-related genes.

Genes in the turquoise and blue modules were enriched by GO and KEGG analyses. GO enrichment analysis of the turquoise module showed that it was mainly enriched to cell cycle processes related to proliferation and metastasis of HCC: BP enrichment resulted in nuclear division, organelle fission, and mitotic nuclear division; CC enrichment results in condensed chromosome, chromosomal region, chromosomal, and centromeric region; MF enrichment results in DNA-dependent ATPase activity (KEGG enrichment results in cell cycle (cell cycle), DNA replication (DNA replication), and neuroactive ligand-receptor interaction (neuroactive ligand-receptor interaction)). In contrast, the blue module reflects the characteristics of liver function itself; BP enrichment results in organic acid catabolic process, carboxylic acid catabolic process, and small molecule catabolic process; CC enrichment results in mitochondrial matrix, peroxisomal matrix, and microbody lumen; MF enriched heme binding, tetrapyrrole binding, and monooxygenase activity; KEGG enrichment results in leucine and isoleucine degradation, fatty acid degradation, and retinol metabolism (Figure 6). The *p* values of the above enrichment analysis results were <0.05.

### 3.4. PPI Network Construction and Core Gene Extraction

Based on MM values, 2000 genes of turquoise were analyzed by STRING. The degree values were visualized by Network Analyzer of Cytoscape software, and the eight genes with the most significant degree values were screened: PLK1, CDK1, CDC20, CCNB2, CCNB1, CCNA2, BUB1B, and BUB1 (Figure 7). Similarly, PPI analysis of genes from the blue module was performed to screen the six genes with the most significant degree values: CAT, ACADM, EHHADH, AGXT, HMGCS2, and CYP3A4 (Figure 7). Interestingly, the PPI analysis of the blue module contained a network of 10 mitochondrial genes with higher degree values.

### 3.5. Six Networks Were Constructed Based on ENCORI

A total of 114 genes were used in the turquoise module to construct the networks, including 106 genes screened in the turquoise module using |MM| > 0.75 as the criterion and 8 genes obtained by PPI analysis. Three turquoise-related networks were established: a lncRNA-miRNA-mRNA coexpression network consisting of 1 lncRNA, 8 miRNAs, and 10 mRNAs; a lncRNA-RBP-mRNA network consisting of 5 lncRNAs, 121 RNA binding proteins (RBPs), and 18 mRNAs; a RBP-mRNA-Tissue-Disease network consists of 104 RBPs, 13 mRNAs, 14 tissue, and 29 diseases (Figure 8).

A total of 128 genes from the blue module were used to construct the network, including 122 genes (106 lncRNAs and 112 mRNAs) screened by MM > 0.6 and 6 genes obtained by PPI analysis. Three turquoise-related networks were established: the lncRNA-miRNA-mRNA coexpression network consisted of 3 lncRNAs, 22 miRNAs, and 29 mRNAs; the lncRNA-RBP-mRNA network consisted of 4 lncRNAs, 128 RNA binding proteins (RBPs), and 112 mRNAs; the RBP-mRNA-Tissue-Disease network consisted of 48 RBPs, 9 mRNAs, 14 tissue, and 22 diseases (Figure 9).

### 3.6. The ROC Curves Showed the Good Performance of the Prognostic Model

Univariate Cox regression analysis was performed on mRNAs and lncRNAs in all differentially expressed genes, turquoise module, and blue module to explore their relationship with prognosis of hepatocellular carcinoma patients. Among all mRNAs, WISP3 (*p* = 0.01) and STK32B (*p* = 0.022) were screened. The AUC values of 3- and 5-year disease-free survival were 0.775 and 0.769, respectively. Among all lncRNAs, AL359853.1 (*p* = 0.005), AC110285.3 (*p* = 0.025), and FGF14-AS2 (*p* = 0.013) were screened. The AUC values of 3- and 5-year disease-free survival were 0.793 and 0.751, respectively. Among lncRNAs in the turquoise module, FGF14-AS2 (*p* = 0.019) was screened. The AUC values of 3- and 5-year disease-free survival were 0.699 and 0.67, respectively. Among mRNAs in the turquoise module, SOX11 (*p* = 0.014), HOXC8 (*p* = 0.004), GAGE2A (*p* < 0.001), and ETV4 (*p* = 0.016) were screened. The AUC values of 3- and 5-year disease-free survival were 0.85 and 0.801, respectively. Among mRNAs in the blue module, CISH (*p* = 0.001) was screened. The AUC values of 3- and 5-year disease-free survival were 0.826 and 0.834, respectively. The same survival analysis was performed for the core genes PLK1, CDK1, CDC20, CCNB2, CCNB1, CCNA2, BUB1B, and BUB1 of PPI in the turquoise module (Figure 10, Figure 11).

KM survival curves were used to observe the relationship between genes and survival. If the survival curves intersected, landmark analysis was performed. Finally, 11 prognosis-related genes were screened for the first time (*p* < 0.01): WISP3, STK32B, AL359853.1, AC110285.3, FGF14-AS2, HOXC8, GAGE2A, CDK1, CDC20, CCNA2, and BUB1. Higher levels of these genes were associated with poorer prognosis and may be poor prognostic liver cancer factors (Figure 12).

While landmark analysis showed that the higher expression levels of ETV4, SOX11, CCNB2, PLK1, BUB1B, and CCNB1 are the worse prognosis, which may be a poor prognostic factor for hepatocellular carcinoma, the higher expression levels of CISH are the better prognosis, which may be a protective factor for HCC prognosis (Figure 13).

### 3.7. GSEA Analysis Revealed 11 Genes Closely Associated with Cell Cycle and Translation

The median expression values of the survival genes screened were divided into two expression level groups. GSEA was then performed to detect the set of genes enriched in the gene classes of both groups to identify their expression levels and pathway associations. In an analysis, mostly, genes were enriched in cell cycle and protein replication-related pathways (Figure 14), further suggesting that these genes proceed to be associated with survival.

### 3.8. Five Machine Learning Models Demonstrated the Importance of 21 Genes in HCC

Gradient boosting, random forest, support vector machine, logistic regression, and integrated learning of data featuring 21 genes, which include the 15 survival-related mRNAs mentioned above and 6 PPI. The mRNAs belong to blue module are as follows: CAT, ACADM, EHHADH, AGXT, HMGCS2, and CYP3A4. The four models for judging HCC were finally generated through training, testing, and validation (Figure 15). The gradient boosting machine's feature contribution degree bar graph showed that CCNB1, GAGE2A, and CYP3A4 were the more important features for judging HCC (Figure 15(c)). And the bar graph of feature contribution degree of random forest showed that CCNB1, BUB1, and CYP3A4 were the more important features for judging HCC (Figure 15(f)). In all metrics, random forest performed the best, and logistic regression was poor, but all these models reflected good training (Table 3). Therefore, we included them in the integrated learning, which uses a voting mechanism; if the voting ratio is 2 : 2, we use the value of random forest. Finally, the accuracy of the test set was improved to 0.97, the accuracy of the validation set was improved to 0.92, and other metrics were also improved (Table 3).

### 3.9. Key Genes Associated with TP53 Mutations, Promoter Methylation, and Immune Cell Infiltration

TP53 is a frequently mutated gene in many cancers. According to the analysis of the UALCAN database, among these genes in hepatocellular carcinoma, all genes were significantly elevated in TP53-mutated tumors except CIHS, where gene expression was significantly decreased in TP53-mutated tumors (Figure 16).

The methylation level of promoter region is closely related to tumor development. Therefore, we analyzed the methylation levels of the promoter regions of these core genes in hepatocellular carcinoma tissues. We found that the promoter methylation levels of CDK1, BUB1, ETV4, PLK1, WISP3, CCNB2, CISH, CCNB1, CCNA2, and GAGE2A were significantly decreased in hepatocellular carcinoma compared with normal tissues, while the promoter methylation levels of STK32B, SOX11, HOXC8, and BUB1B were significantly increased compared with normal tissues (Figure 17).

We analyzed the relationship between these core genes and immune cell infiltration through the TIMER 2.0 website. The heat map showed that all these genes were associated with immune cell infiltration and were mainly distributed on CD4 T cells, macrophage, regulatory T cells, and monocyte. As a whole, these genes clustered into two different parts, and their relationship with immune cell infiltration was almost completely opposite. The clustering results also showed that these genes could be divided into two clusters. The first cluster contains ACADM, AGXT, CAT, CISH, CYP3A4, EHHADH, FGF14-AS2, HMGCS2, and WISP3 genes, which are negatively associated with CD4 T cells, macrophages, and regulatory T cells, and positively associated with monocytes. Interestingly, in addition to the seven genes in the blue module, WISP3 and FGF14-AS2 in the turquoise module were also clustered in the first cluster and were clustered together. The second cluster is almost the exact opposite of the first cluster in terms of immune cell infiltration relationship (Figure 18). The correlation between them was further confirmed by the relationship map between genes (Figure 19).

KEGG pathway enrichment showed that the first cluster was mainly metabolism-related pathways, and since the previous machine learning results showed that CYP3A4 was an important feature-contributing gene in the hepatocellular carcinoma diagnostic model, we expanded the *p* adjust value to 0.56 to include linoleic acid metabolism (LAM) containing CYP3A4 as a pathway of interest, in addition to some pathways of metabolism, PPAR signaling pathway, and terpenoid backbone biosynthesis. In the second cluster, besides cell cycle-related pathways, progesterone-mediated oocyte maturation, p53 signaling pathway, FOXO signaling pathway, and immune abnormalities-related pathways were also enriched (Figure 20).

### 3.10. Screening and Molecular Docking of Four Gene Candidates

Proteins without structure in the RCSB PDB library were excluded. A total of 257 small molecules related to CCNA2, CCNB1, CDK1, and PLK1 with high feature contribution in machine learning were obtained by DGIdb online tool. The PDB structure 2IW8 for CCNA2, 4YC3 for CCNB1, 6GU6 for CDK1, and 3DB6 for PLK1 were obtained from the RCSB PDB library were obtained. Under the condition of docking affinity score greater than -7.0 kcal/mol, 8 small molecules were found to have high affinity with cyclin A2 expressed by CCNA2, 44 small molecules had high affinity with G2/mitotic-specific cyclin-B1 expressed by CCNB1, 184 small molecules had high affinity to CDK1-expressed cyclin-dependent kinase 1 (CDK1), and 191 small molecules had high affinity to PLK1-expressed polo-like kinase 1 (PLK1) (Table 4). Among them, ZINC40393428, ZINC3973984, and ZINC20149014 had high affinity in all four (Figure 21).

## 4. Discussion

HCC is a high mortality disease among cancers worldwide and has a poor prognosis. Not all patients are suitable for surgical treatment [34]. Alpha-fetoprotein (AFP) is a tumor marker secreted by different levels of hepatocellular carcinoma and therefore is often used as one of the few means to detect hepatocellular carcinoma [35]. However, some literature suggests that it is controversial [36–38]. Competitive binding to miRNA in lncRNA-miRNA-mRNA plays an important role in cancer development and regulation [39, 40]. We obtained turquoise and blue modules by WGCNA. Pathway analysis showed that the turquoise module is associated with cell cycle and DNA replication, and the blue module is mostly distributed in metabolism-related pathways. Accordingly, the ceRNA networks of both were constructed. Many of these genes have been shown to be associated with liver cancer. For example, in the turquoise module, the SNHG1 gene has been shown to be involved in cancer regulation, including hepatocellular carcinoma, through multiple ceRNA pathways [41]. The lncRNA-RBP-mRNA network was also constructed based on the theory that lncRNA recruitment of RBP affects mRNA [42]. Interestingly, SNHG1 was still included. We constructed an RBP-mRNA-Tissue-Disease network and showed that these combinations are frequently found in breast and liver and are mostly malignant epithelial tumors. Indeed, breast cancer has a very subtle relationship with the liver [43]. The results of our study also confirm the existence of this close relationship.

By univariate—Lasso—multiple Cox regression analysis and PPI, we obtained 11 genes according to survival time: WISP3, STK32B, AL359853.1, AC110285.3, FGF14-AS2, HOXC8, GAGE2A, CDK1, CDC20, CCNA2, and BUB1. These genes may be associated with prognostic relevance. WISP3 is a member of the CCN family, a family of cysteine-rich glycosylated proteins that are expressed in development and disease onset [44]. The results of our survival analysis were similar to other results where survival curves showed it to be a poor prognostic factor for hepatocellular carcinoma [45]. However, some studies have reported that WISP3 has the potential to inhibit the development of hepatocellular carcinoma [46–48]. Indeed, the role of WISP3 seems to be different in different cancers [49], suggesting its complex regulatory mechanisms. STK32B is mainly associated with idiopathic tremor and anxiety [50, 51], but Parris et al. found that it may be a marker for oral squamous cell carcinoma [52]. AL359853.1, AC110285.3, and GAGE2 have also been noted to be possibly associated with the prognosis of HCC [53–55]. HOXC8 is a potential driver gene for many cancer cells and is associated with cell proliferation, adhesion, migration, and metabolism-related processes and can be considered as a global regulator of growth and differentiation [56–59]. FGF14-AS2 has inhibitory effects on breast and colorectal cancers [60, 61] but has a promotive effect on gliomas [62], and its role in hepatocellular carcinoma has not been reported. CDK1 is required for mammalian cell proliferation. It is the only CDK that can initiate mitosis (i.e., M phase) [63], but tumor cells may also require specific interphase CDKs to proliferate. Therefore, selective CDK inhibition may provide therapeutic benefit in some human tumors [64]. CDC20 exerts its biological functions mainly by targeting its downstream substrates for ubiquitination and subsequent degradation [65] and plays a role in the cell cycle and apoptosis [66, 67]. In hepatocellular carcinoma, inhibition of CDC20 decreases cell proliferation in hepatocellular carcinoma cells [68]. CDC20 acts by various mechanisms, such as involvement in the p53-related pathway [69]. Ubiquitination of CCNA2 is associated with CDC20; the late promotion complex of ubiquitinated CCNA2 is activated by CDC20 [70], and its overexpression is frequently observed in hepatocellular carcinoma [71] and is a more recognized marker [72]. The spindle assembly checkpoint is an important monitoring mechanism to ensure high-fidelity mitotic chromosome segregation. This is achieved by monitoring whether sister chromatids lack tension or are attached to spindle microtubules. It is mediated by checkpoint complexes or individual proteins that inhibit late promoting complex/loop (APC/C) ubiquitin ligase activity by targeting CDC20 regulatory subunits. BUB1 kinase is a key spindle checkpoint regulatory protein [73]. BUB1 may promote proliferation of hepatocellular carcinoma cells by activating phosphorylation of SMAD2 [74]. Not surprisingly, among them, CDC20, CCNA2, and BUB1 are all associated with APC-related processes, which may be key nodes in the prognosis and occurrence of hepatocellular carcinoma. GSEA enrichment results suggest that these genes are associated with replication, translation, and chromosome formation.

To improve the accuracy and enrich the means of hepatocellular carcinoma diagnosis, we performed integrated learning to build a hepatocellular carcinoma discriminative model using the core genetic composition features of the survival time module and other modules with higher span and tried to improve the diagnosis rate by machine learning, and the results showed that our model had high accuracy and AUC value.

In general, predictions are mainly based on the compositional features of genes and metabolites [75, 76]. CCNB1 is the gene with a large feature contribution in the model. During cytokinesis, CCNB1 binds to CDK1 to transition the cell from G2 phase to mitosis. After mid mitosis, cell cycle proteins are separated from CDK, and in the presence of APC, M phase cyclin A and cyclin B are degraded by the proteasome through ubiquitination-dependent pathway [75], and CCNB1 is also known to promote cancer development [76]. PLK1 is an inhibitor of the regulatory late promoting complex/cyclosome (APC/C) and can synergistically promote cell cycle protein B/Cdk1-mediated APC/C activation [77].

These related genes obtained by analysis of TP53 mutations, promoter methylation, and immune cell infiltration influence the progression of hepatocellular carcinoma in these aspects. By looking at the clustering results from an immune perspective, it is easy to distinguish between the blue module and other genes outside of it. And the results of KEGG pathway analysis also suggest that these core genes are involved in some immune-related pathways.

Recent studies have shown that dysregulation of propionate metabolism produces a prometastatic profile in breast and lung cancer cells, promoting cancer progression [78]. In contrast, linoleic acid and butyric acid have therapeutic potential for cancer, and they are both implicated in intestinal flora metabolism [79, 80], and intestinal flora and related metabolite molecules, which translocate through the portal vein to the liver and affect liver function, portend a potential pathway for intestinal flora to treat liver cancer. Peroxisome proliferator-activated receptor (PPAR) belongs to a class of nuclear hormone receptors activated by fatty acids and their derivatives, which have been shown to have cell cycle and metabolic regulatory effects. Some evidence suggests that it has a promotive effect on hepatocellular carcinoma and can be used as a target for drugs [81, 82].

Branched-chain amino acid metabolism is the most significant pathway obtained in the analysis, and studies have shown that the supplementation of valine, leucine, and isoleucine in branched-chain amino acids has a preventive effect on hepatocellular carcinoma [83]. In cluster II, in addition to the pathways of senescence and cell proliferation that often accompany cancer, we identified two interesting pathways—the progesterone-mediated oocyte maturation pathway and the oocyte meiotic pathway.

Although the role of progesterone-mediated oocyte maturation pathway and oocyte meiosis pathway in hepatocellular carcinoma is not clear, it has been reported in the literature that glioblastoma, lung cancer, etc. appear to be genetically enriched in these two pathways [84, 85]. Hepatocellular carcinoma is a sex-specific cancer, and in general, men are two to four times more likely to develop HCC than women [86], which predicts that some hormonal changes may contribute to this difference, among which progesterone receptor expression can affect the proliferation of hepatocellular carcinoma [87]. Enriched pathway, in which the FOXO transcription factor family plays an important role in tumor proliferation and apoptosis [88], FOXO1 was shown to play a repressive role in hepatocellular carcinoma [89], and other FOXO transcription factors have been shown to be associated with hepatocellular carcinoma [90, 91]. These evidences suggest that the genes we screened affect the progression of hepatocellular carcinoma by influencing the metabolic, immune, and other pathways.

Finally, we screened for potential drug candidates that might have an effect on HCC. To our surprise, many of these drugs have been found to have therapeutic effects on hepatocellular carcinoma, although the association with the genes we identified is not yet clear. For example, ZINC9566782 (hygromycin) has the highest docking affinity for cyclin A2. It suppresses stemness and malignancy of HCC cells by destroying CD133 in the LCSC population [92]. ZINC40393428 (SNS-314) has also been shown to be efficacious in hepatocellular carcinoma [93]. Our study provides recommendations for the diagnosis and treatment of hepatocellular carcinoma. However, due to the limitations of TCGA and GEO libraries, our results may need to be demonstrated by follow-up experiments.

Only a few machine learning algorithms are used in this study. In addition to the methods used in this paper, some of the most representative computational intelligence algorithms can be used to solve the problem, such as monarch butterfly optimization (MBO), earthworm optimization algorithm (EWA), elephant herding optimization (EHO), moth search (MS) algorithm, slime mold algorithm (SMA), hunger games search (HGS), Runge Kutta optimizer (RUN), colony predation algorithm (CPA), and Harris hawks optimization (HHO). These algorithms have the potential to provide better choices for our models. Many learning techniques have been developed to improve the performance of metaheuristic algorithms, such as the dynamic learning evolution algorithm (DLEA) [94] and the learning-based intelligent optimization algorithm (LIOA) [95]. This may be another effective way to improve model performance, and we will consider them in our subsequent studies. In addition, some biological experiments are also worth drawing on to demonstrate the reliability of the model and the importance of biomarkers [96].

## 5. Conclusions

In conclusion, we screened 2 modules, 6 networks, and 24 genes for hepatocellular carcinoma. Five machine learning models were constructed and screened for drug candidates for the core genes. This suggests that hepatocarcinogenesis is a dynamic network with multiple mechanisms. Treating only one pathway or one type of gene is not appropriate, especially since the liver is involved in various metabolic pathways. Combining dynamic therapies may be the hope for a complete cure of liver cancer in the future.

## Figures and Tables

**Figure 1:** Overall flowchart of this study.

**Figure 2:** Differential analysis of data in the TCGA-LIHC samples. The volcano map for differential genes is presented, in which the *x*-axis represents −log10 (FDR), and the *y*-axis represents logFC. Each dot in the map represents a gene, where the red dots represent the upregulated genes in HCC, and the blue dots represent the downregulated genes in HCC: (a) lncRNA, (b) mRNA, and (c) miRNA.

**Figure 3:** GO and KEGG pathway analyses of upregulated and downregulated differential mRNA. (a) GO biological process (GO-BP) of upregulated differential mRNA. (b) GO cellular component (GO-CC) of upregulated differential mRNA. (c) GO molecular function (GO-MF) of upregulated differential mRNA. (d) KEGG pathway of upregulated differential mRNA. (e) GO-BP of downregulated differential mRNA. (f) GO-CC of downregulated differential mRNA. (g) GO-MF of downregulated differential mRNA. (h) KEGG pathway of downregulated differential mRNA.

**Figure 4:** (a) Multivariate Cox regression forest map. (b) ROC curve used to evaluate prognosis model. (c) KM curve of total bilirubin upper limit. (d) KM curve of prognostic genes combined with landmark analysis.

**Figure 5:** (a) Power value screening by WGCNA. (b) Module-feature correlation. Each row corresponds to a module, and each column corresponds to a feature, including the corresponding correlation and *p* value. The characteristics represented by letters are (A) age at initial pathological diagnosis, (B) bilirubin lower limit, (C) bilirubin upper limit, (D) surv time, (E) fetoprotein output value, and (F) total bilirubin upper limit. (c) Module characteristic gene clustering heat map. (d) Tom diagram in the module. Dark color indicates topological overlap, and light color indicates high topological overlap.

**Figure 6:** (a) GO biological process (GO-BP) of turquoise modules. (b) GO cellular component (GO-CC) of turquoise modules. (c) GO molecular function (GO-MF) of turquoise modules. (d) KEGG pathway of turquoise modules. (e) GO-BP of blue modules. (f) GO-CC of blue modules. (g) GO-MF of blue modules. (h) KEGG pathway of blue modules.

**Figure 7:** (a) The PPI network diagram of the first 2000 genes of turquoise module. (b) The PPI network diagram of blue module. The darker the color and the larger the shape mean, the greater the degree contribution.

**Figure 8:** Network diagram of turquoise module with |MM| > 0.75 and its PPI hub gene; the darker the color, the larger the shape, representing a greater degree contribution. (a) Coexpression network of lncRNA-miRNA-mRNA: the hub lncRNA is SNHG1; the hub of miRNA is hsa-miR-3918; the hubs of mRNAs are MCM8 and PHF19. (b) lncRNA-RBP-mRNA network: the hub lncRNAs are SNHG1 and LENG8-AS1; the hub RBPs are SRSF1 and EIF4A3; the hub mRNAs are BUB1, RBL1, and KIF18B. (c) RBP-mRNA-Tissue-Disease network: hub RBPs are IGF2BP2 and EIF4A3; hub mRNAs are PLK1and CDC20; hub organs are breast and liver; hub disease is carcinoma.

**Figure 9:** Network diagram of blue module with |MM| > 0.6 and its PPI hub gene: the darker the color, the larger the shape, representing a greater degree contribution. (a) Coexpression network of lncRNA-miRNA-mRNA: the hub lncRNAs are LINC00261 and DHRS4-AS1; the hubs of miRNAs are hsa-miR-1270 and hsa-miR-2278; the hub of mRNA is ATP11C. (b) lncRNA-RBP-mRNA network: the hub lncRNAs are LINC00261 and LINC01018; the hub RBPs are FUS and TAF15; the hub mRNAs are MTHFD1 and LARP1B. (c) RBP-mRNA-Tissue-Disease network: hub RBPs are EIF4A3 and IGF2BP2; hub mRNAs are MTHFD1 and AL139011.2; hub organs are breast and liver; hub disease is carcinoma.

**Figure 10:** Left: characteristic influencing factor model penalty process. Right: optimal penalty coefficient in Lasso regression model *λ* change process. (a) All mRNA.(b) All lncRNA. (c) lncRNA of turquoise module. (d) mRNA of turquoise module. (e) mRNA of blue module.

**Figure 11:** Lasso and multiple Cox regression analysis results. Left: Cox regression analysis results forest map. Middle: ROC curve was used to evaluate the prognosis model. Right: KM curve of risk level. (a) All mRNA. (b) All lncRNA. (c) lncRNA of turquoise module. (d) mRNA of turquoise module. (e) mRNA of blue module.

**Figure 12:** KM curve of 11 prognostic genes: (a) STK32B, (b) WISP3, (c) FGF14-AS2, (d) CCNA2, (e) AL359853.1, (f) AC110285.3, (g) HOXC8, (h) GAGE2A, (i) BUB1, (j) CDK1, and (k) CDC20.

**Figure 13:** KM curve after Cox analysis (left). KM curve of prognostic gene after landmark analysis (right). (a) BUB1B. (b) PLK1. (c) SOX11. (d) ETV4. (e) CISH. (f) CCNB2. (g) CCNB1.

**Figure 14:** GSEA pathway analysis of 11 genes.

**Figure 15:** (a) ROC curve of gradient boosting test set (AUC > 0.966). (b) ROC curve of gradient boosting verification set (AUC > 0.926). (c) The feature importance of gradient boosting training concentration. (d) ROC curve of random forest test set (AUC > 0.967). (e) ROC curve of random forest validation set (AUC > 0.937). (f) Characteristic importance of random forest training set. (g) ROC curve of support vector machine test set (AUC > 0.966). (h) ROC curve of support vector machine validation set (AUC > 0.948). (i) ROC curve of logistic regression test set (AUC > 0.927). (j) ROC curve of logistic regression validation set (AUC > 0.946).

**Figure 16:** Relationship between hub RNA expression and TP53 mutation: (a) CDK1; (b) STK32B; (c) SOX11; (d) BUB1; (e) CDC20; (f) ETV4; (g) PLK1; (h) WISP3; (i) CCNB2; (j) CISH; (k) HOXC8; (l) BUB1B; (m) CCNB1; (n) CCNA2.

**Figure 17:** Relationship between hub RNA expression and promoter methylation: (a) CDK1; (b) STK32B; (c) SOX11; (d) BUB1; (e) CDC20; (f) ETV4; (g) PLK1; (h) WISP3; (i) CCNB2; (j) CISH; (k) HOXC8; (l) BUB1B; (m) CCNB1; (n) CCNA2; (o) GAGE2A.

**Figure 18:** Heat map of the correlation between immune cell infiltration predicted by six algorithms and hub gene expression: (a) CIBERSORT; (b) CIBERSORT.ABS; (c) xCell; (d) TIMER; (e) quanTIseq; (f) EPIC.

**Figure 19:** Heat map of the relationship in hub genes.

**Figure 20:** KEGG pathway analysis of hub genes. (a) KEGG pathway bar chart for cluster one gene. (b) KEGG network diagram of cluster one gene. (c) KEGG pathway bar chart for cluster two genes. (d) KEGG network diagram of cluster two genes.

**Figure 21:** The result of candidate drugs with the highest affinity (left), ZINC40393428, ZINC3973984, and ZINC20149014 (right) docked with four PDB structures. (a) Docking results of ZINC95626782 with cyclin A2. (b) The docking results of ZINC40393428, ZINC3973984, and ZINC20149014 with cyclin A2 are arranged from left to right. (c) Docking results of ZINC3817327 with G2/mitotic-specific cyclin-B1. (d) The docking results of ZINC40393428, ZINC3973984, and ZINC20149014 with G2/mitotic-specific cyclin-B1 are arranged from left to right. (e) Docking results of ZINC13597410 with cyclin-dependent kinase 1. (f) The docking results of ZINC40393428, ZINC3973984, and ZINC20149014 with cyclin-dependent kinase 1 are arranged from left to right. (g) Docking results of ZINC9407473 with polo-like kinase 1. (h) The docking results of ZINC40393428, ZINC3973984, and ZINC20149014 with polo-like kinase 1 are arranged from left to right.

**Table 1:** Univariate Cox regression results.

Clinical	HR	*P*
Total_bilirubin_upper_limit	35.41655389	3.31E-07
Platelet_result_lower_limit	1.070080085	0.006911203
Platelet_result_upper_limit	1.068948854	0.008341265
Platelet_result_count	1.051063842	0.059517343
Neoplasm_histologic_grade	1.250333525	0.127362381
Fetoprotein_outcome_value	0.977247772	0.162204753
Weight	0.772356088	0.208050661
Age_at_initial_pathologic_diagnosis	0.859880674	0.453564629
Sample_type	0.47341456	0.456630015
Bilirubin_lower_limit	0.604438968	0.474436464
Gender	0.936796253	0.67689342
Bilirubin_upper_limit	0.964460012	0.814065126
Histological_type	0.859604808	0.854789298

**Table 2:** Gene number of each module in WGCNA.

Module	Number
Tan	55
Black	115
Blue	561
Cyan	47
Green yellow	57
Red	178
Yellow	208
Grey60	36
Light green	36
Light yellow	33
Royal Blue	32
Light cyan	37
Brown	409
Magenta	84
Salmon	49
Green	181
Purple	60
Turquoise	3174
Midnight blue	45
Pink	114
Grey	989

**Table 3:** Training effects of five models: 0 is a normal sample, and 1 is a cancer sample.

Model	Set	Indicators				
Gradient boosting	5-fold cross-validation	0.91397849	0.93548387	0.9673913	0.95652174	0.95652174
	Leave-one-out method	Mean accuracy: 0.94				
	Test set		Precision	Recall	f1-score	Support
		0	0.88	0.85	0.86	26
		1	0.96	0.97	0.96	90
		Accuracy			0.94	116
		Macro average	0.92	0.91	0.91	116
		Weighted average	0.94	0.94	0.94	116
	Validation set (default value)		Precision	Recall	f1-score	Support
		0	0.88	0.89	0.88	105
		1	0.92	0.91	0.92	152
		Accuracy			0.90	257
		Macro average	0.90	0.90	0.90	257
		Weighted average	0.90	0.90	0.90	257

Random forest	5-fold cross-validation	0.93548387	0.95698925	0.97826087	0.97826087	0.9673913
	Leave-one-out method	Mean accuracy:0.96				
	Test set		Precision	Recall	f1-score	Support
		0	0.92	0.88	0.90	26
		1	0.97	0.98	0.97	90
		Accuracy			0.96	116
		Macro average	0.94	0.93	0.94	116
		Weighted average	0.96	0.96	0.96	116
	Validation set (threshold = 0.4)		Precision	Recall	f1-score	Support
		0	0.93	0.85	0.89	105
		1	0.90	0.95	0.93	152
		Accuracy			0.91	257
		Macro average	0.91	0.90	0.91	257
		Weighted average	0.91	0.91	0.91	257

SVM	5-fold cross-validation	0.90322581	0.91397849	0.93478261	0.93478261	0.91304348
	Leave-one-out method	Mean accuracy:0.91				
	Test set		Precision	Recall	f1-score	Support
		0	0.74	0.88	0.81	26
		1	0.96	0.91	0.94	90
		Accuracy			0.91	116
		Macro average	0.85	0.90	0.87	116
		Weighted average	0.91	0.91	0.91	116
	Validation set (default value)		Precision	Recall	f1-score	Support
		0	0.91	0.85	0.88	105
		1	0.90	0.94	0.92	152
		Accuracy			0.90	257
		Macro average	0.90	0.89	0.90	257
		Weighted average	0.90	0.90	0.90	257

Logistic Regression	5-fold cross-validation	0.91397849	0.93548387	0.89130435	0.94565217	0.91304348
	Leave-one-out method	Mean accuracy:0.91				
	Test set		Precision	Recall	f1-score	Support
		0	0.76	0.85	0.80	26
		1	0.95	0.92	0.94	90
		Accuracy			0.91	116
		Macro average	0.86	0.88	0.87	116
		Weighted average	0.91	0.91	0.91	116
	Validation set (default value)		Precision	Recall	f1-score	Support
		0	0.88	0.80	0.84	105
		1	0.87	0.93	0.90	152
		Accuracy			0.88	257
		Macro average	0.88	0.86	0.87	257
		Weighted average	0.88	0.88	0.87	257

Integrated learning	Test set		Precision	Recall	f1-score	Support
		0	0.96	0.92	0.94	26
		1	0.98	0.99	0.98	90
		Accuracy			0.97	116
		Macro average	0.97	0.96	0.96	116
		Weighted average	0.97	0.97	0.97	116
	Validation set		Precision	Recall	f1-score	Support
		0	0.90	0.90	0.90	105
		1	0.90	0.95	0.93	152
		Accuracy			0.92	257
		Macro average	0.92	0.92	0.92	257
		Weighted average	0.92	0.92	0.92	257

**Table 4:** Docking results of four proteins with molecules in small molecule library (candidate drug list).

Cyclin A2		G2/mitotic-specific cyclin-B1		Cyclin-dependent kinase 1		Polo-like kinase 1	
Molecule	Affinity	Molecule	Affinity	Molecule	Affinity	Molecule	Affinity
ZINC95626782	-7.6	ZINC3817327	-8.9	ZINC13597410	-10.1	ZINC9407473	-10.7
ZINC9495236	-7.6	ZINC3973984	-8.4	ZINC100461551	-10	ZINC43203898	-10.1
ZINC1629864	-7.4	ZINC3814435	-8.2	ZINC3939511	-9.7	ZINC43128366	-10
ZINC40393428	-7.2	ZINC5328058	-8.1	ZINC35930738	-9.6	ZINC21288966	-9.9
ZINC3817327	-7.1	ZINC3879185	-7.7	ZINC23894	-9.6	ZINC40393428	-9.7
ZINC3973984	-7	ZINC3920266	-7.7	ZINC1554668	-9.6	ZINC34638188	-9.6
ZINC14948097	-7	ZINC3861470	-7.7	ZINC29053046	-9.5	ZINC34285229	-9.6
ZINC20149014	-7	ZINC1554668	-7.6	ZINC2109876	-9.3	ZINC34285233	-9.6
		ZINC43154472	-7.6	ZINC3780893	-9.3	ZINC340372	-9.6
		ZINC100461551	-7.5	ZINC3817793	-9.3	ZINC3939511	-9.5
		ZINC100001998	-7.5	ZINC43154472	-9.2	ZINC25958	-9.5
		ZINC34285229	-7.5	ZINC851497	-9.2	ZINC64373300	-9.5
		ZINC3986640	-7.4	ZINC34285229	-9.2	ZINC3820327	-9.4
		ZINC35930738	-7.4	ZINC100001998	-9.2	ZINC1621536	-9.4
		ZINC538152	-7.3	ZINC3872446	-9.2	ZINC29053046	-9.4
		ZINC3861600	-7.3	ZINC21673413	-9.2	ZINC43196885	-9.4
		ZINC13597410	-7.3	ZINC5765083	-9.1	ZINC538152	-9.4
		ZINC34948948	-7.3	ZINC5597201	-9.1	ZINC6745792	-9.4
		ZINC5597201	-7.3	ZINC8829745	-9.1	ZINC2109876	-9.4
		ZINC43128366	-7.3	ZINC34285233	-9.1	ZINC14948097	-9.4
		ZINC49785138	-7.3	ZINC3820327	-9.1	ZINC3995991	-9.3
		ZINC3820327	-7.3	ZINC1639355	-9.1	ZINC21983587	-9.3
		ZINC1621536	-7.2	ZINC34894449	-9	ZINC3817327	-9.2
		ZINC43196885	-7.2	ZINC49785138	-9	ZINC3817793	-9.2
		ZINC3860715	-7.2	ZINC3954595	-9	ZINC16052807	-9.2
		ZINC8762246	-7.2	ZINC34948948	-8.9	ZINC3830466	-9.1
		ZINC34285233	-7.2	ZINC3879185	-8.9	ZINC14963227	-9.1
		ZINC9073	-7.2	ZINC14945777	-8.9	ZINC37868887	-9.1
		ZINC4822288	-7.2	ZINC72107868	-8.9	ZINC43154472	-9.1
		ZINC2109876	-7.2	ZINC20149024	-8.9	ZINC49785138	-9.1
		ZINC21288966	-7.2	ZINC9073	-8.9	ZINC20149014	-9.1
		ZINC20533312	-7.1	ZINC21288966	-8.9	ZINC3941269	-9.1
		ZINC34894449	-7.1	ZINC19632891	-8.8	ZINC3986640	-9
		ZINC5765083	-7.1	ZINC4822288	-8.8	ZINC13597410	-9
		ZINC4543798	-7.1	ZINC100706870	-8.8	ZINC3029819	-9
		ZINC12726360	-7.1	ZINC8681123	-8.8	ZINC236195	-9
		ZINC1619592	-7.1	ZINC538152	-8.8	ZINC602090	-9
		ZINC3939511	-7.1	ZINC1559601	-8.8	ZINC34948948	-9
		ZINC3941269	-7.1	ZINC5582530	-8.8	ZINC100001998	-9
		ZINC8829745	-7.1	ZINC21983587	-8.8	ZINC13121831	-8.9
		ZINC4817100	-7	ZINC3815419	-8.8	ZINC20533312	-8.9
		ZINC40393428	-7	ZINC43196885	-8.6	ZINC3920266	-8.9
		ZINC20149014	-7	ZINC9331709	-8.6	ZINC1487934	-8.9
		ZINC169335484	-7	ZINC16052807	-8.6	ZINC4822288	-8.9
				ZINC1841840	-8.6	ZINC3879185	-8.9
				ZINC14948097	-8.6	ZINC49113058	-8.9
				ZINC3861633	-8.6	ZINC4976875	-8.9
				ZINC20149014	-8.5	ZINC100235333	-8.9
				ZINC1629864	-8.5	ZINC196663	-8.8
				ZINC12726360	-8.5	ZINC599734	-8.8
				ZINC155803	-8.5	ZINC20149017	-8.8
				ZINC1700953	-8.5	ZINC8762246	-8.8
				ZINC20149017	-8.5	ZINC3973984	-8.8
				ZINC16052674	-8.4	ZINC5328058	-8.8
				ZINC13340605	-8.4	ZINC9495236	-8.8
				ZINC16052857	-8.4	ZINC72107868	-8.8
				ZINC1649340	-8.4	ZINC8829745	-8.8
				ZINC1621536	-8.4	ZINC16052682	-8.7
				ZINC1606505	-8.4	ZINC53119602	-8.7
				ZINC49113058	-8.4	ZINC1629864	-8.7
				ZINC25958	-8.4	ZINC100461551	-8.7
				ZINC4016162	-8.4	ZINC100706870	-8.7
				ZINC37868887	-8.4	ZINC4817100	-8.7
				ZINC4475360	-8.4	ZINC5247757	-8.7
				ZINC1689786	-8.4	ZINC8681123	-8.7
				ZINC602192	-8.4	ZINC3842402	-8.6
				ZINC12504456	-8.4	ZINC4015433	-8.6
				ZINC3986640	-8.4	ZINC3814435	-8.6
				ZINC6745792	-8.4	ZINC38698888	-8.6
				ZINC340372	-8.4	ZINC9331709	-8.6
				ZINC6514705	-8.4	ZINC18825330	-8.6
				ZINC39001795	-8.3	ZINC1554668	-8.6
				ZINC599734	-8.3	ZINC3873287	-8.6
				ZINC4015433	-8.3	ZINC3798734	-8.6
				ZINC2002752	-8.3	ZINC12726360	-8.6
				ZINC1904	-8.3	ZINC2047389	-8.6
				ZINC34638188	-8.2	ZINC3861633	-8.5
				ZINC20533312	-8.2	ZINC1559601	-8.5
				ZINC3029819	-8.2	ZINC5597201	-8.5
				ZINC18825330	-8.2	ZINC4693574	-8.5
				ZINC16052682	-8.2	ZINC75148	-8.5
				ZINC1853550	-8.2	ZINC6514705	-8.5
				ZINC608205	-8.2	ZINC5582530	-8.5
				ZINC3938688	-8.2	ZINC3273193	-8.5
				ZINC21486914	-8.2	ZINC16052857	-8.4
				ZINC3873287	-8.2	ZINC16186602	-8.4
				ZINC3995991	-8.1	ZINC1841840	-8.4
				ZINC196663	-8.1	ZINC3356648	-8.4
				ZINC17175232	-8.1	ZINC1687300	-8.4
				ZINC4817100	-8.1	ZINC1687273	-8.4
				ZINC3842402	-8.1	ZINC3988917	-8.4
				ZINC1066512	-8.1	ZINC549484	-8.3
				ZINC3973984	-8.1	ZINC3872446	-8.3
				ZINC9407473	-8.1	ZINC4762361	-8.3
				ZINC3988917	-8.1	ZINC19632891	-8.3
				ZINC14963227	-8.1	ZINC41714	-8.3
				ZINC75148	-8.1	ZINC55760827	-8.3
				ZINC13130211	-8.1	ZINC386389	-8.2
				ZINC3816409	-8	ZINC23894	-8.2
				ZINC4976875	-8	ZINC5765083	-8.2
				ZINC1487934	-8	ZINC9073	-8.2
				ZINC584092	-8	ZINC678019	-8.2
				ZINC52509437	-8	ZINC13983251	-8.2
				ZINC1687300	-8	ZINC1619592	-8.2
				ZINC4822587	-8	ZINC4543798	-8.2
				ZINC2990483	-8	ZINC13340605	-8.1
				ZINC678019	-8	ZINC3815419	-8.1
				ZINC2047389	-7.9	ZINC34894449	-8.1
				ZINC3356648	-7.9	ZINC4016162	-8.1
				ZINC13121831	-7.9	ZINC21673413	-8.1
				ZINC37868756	-7.9	ZINC4475360	-8.1
				ZINC549484	-7.9	ZINC3830394	-8
				ZINC27999611	-7.9	ZINC4822587	-8
				ZINC1697899	-7.9	ZINC851497	-8
				ZINC1687273	-7.8	ZINC3816409	-8
				ZINC40393428	-7.8	ZINC95626782	-8
				ZINC3273193	-7.8	ZINC13986815	-8
				ZINC43131420	-7.8	ZINC584092	-8
				ZINC1670146	-7.8	ZINC3812869	-7.9
				ZINC4762361	-7.8	ZINC4903379	-7.9
				ZINC4543798	-7.8	ZINC155803	-7.9
				ZINC1530689	-7.7	ZINC602192	-7.9
				ZINC16052675	-7.7	ZINC1066512	-7.9
				ZINC4903379	-7.7	ZINC1473	-7.9
				ZINC43128366	-7.7	ZINC52509437	-7.9
				ZINC3886406	-7.7	ZINC3874317	-7.9
				ZINC16052718	-7.7	ZINC608205	-7.9
				ZINC3798734	-7.7	ZINC1904	-7.9
				ZINC8214597	-7.7	ZINC3873285	-7.9
				ZINC3814435	-7.7	ZINC2665575	-7.8
				ZINC1554390	-7.7	ZINC44953	-7.8
				ZINC386389	-7.7	ZINC1649340	-7.8
				ZINC1757986	-7.6	ZINC3860715	-7.8
				ZINC40442496	-7.6	ZINC3861470	-7.8
				ZINC3918156	-7.6	ZINC39001795	-7.8
				ZINC603047	-7.6	ZINC40442496	-7.8
				ZINC14806879	-7.6	ZINC3938688	-7.8
				ZINC340306	-7.6	ZINC603047	-7.8
				ZINC3874317	-7.6	ZINC1700953	-7.8
				ZINC2665575	-7.6	ZINC1606505	-7.8
				ZINC3775641	-7.5	Ebselen	-7.8
				ZINC3878528	-7.5	ZINC14945777	-7.8
				ZINC294736	-7.5	ZINC3954595	-7.7
				ZINC13132551	-7.5	ZINC275332	-7.7
				ZINC44953	-7.5	ZINC3918156	-7.7
				ZINC38698888	-7.5	ZINC3950132	-7.7
				ZINC225430	-7.5	ZINC1639355	-7.7
				ZINC20149019	-7.5	ZINC20149024	-7.7
				ZINC3873285	-7.5	ZINC169335484	-7.7
				ZINC41714	-7.4	ZINC2139624	-7.6
				ZINC1473	-7.4	ZINC3780893	-7.6
				ZINC4693574	-7.4	ZINC14806879	-7.6
				ZINC13983251	-7.4	ZINC8214597	-7.6
				ZINC3950132	-7.4	ZINC3775641	-7.6
				ZINC4411063	-7.4	ZINC340306	-7.6
				ZINC233343	-7.3	ZINC225430	-7.6
				ZINC3830394	-7.3	ZINC1697899	-7.6
				Ebselen	-7.3	ZINC2002752	-7.5
				ZINC5247757	-7.3	ZINC4411063	-7.5
				ZINC3812869	-7.3	ZINC294736	-7.5
				ZINC1530968	-7.3	ZINC13130211	-7.5
				ZINC8035014	-7.3	ZINC237953	-7.5
				ZINC4707792	-7.3	ZINC43131420	-7.5
				ZINC1531764	-7.2	ZINC1722140	-7.5
				ZINC236195	-7.2	ZINC16052718	-7.5
				ZINC602090	-7.2	ZINC4707792	-7.5
				ZINC13514886	-7.2	ZINC643046	-7.5
				ZINC1722140	-7.2	ZINC20149019	-7.5
				ZINC16186602	-7.2	ZINC85534336	-7.5
				ZINC4009000	-7.2	ZINC3886406	-7.4
				ZINC64373300	-7.2	ZINC37868756	-7.4
				ZINC4183729	-7.2	ZINC1531764	-7.3
				ZINC2139624	-7.2	ZINC8035014	-7.3
				ZINC1619592	-7.2	ZINC21486914	-7.3
				ZINC137884	-7.2	ZINC1757986	-7.3
				ZINC9495236	-7.1	ZINC3942646	-7.3
				ZINC388510	-7.1	ZINC13132551	-7.3
				ZINC13571422	-7.1	ZINC12474579	-7.3
				ZINC237953	-7	ZINC3878528	-7.2
				ZINC100037272	-7	ZINC1530968	-7.2
				ZINC3942646	-7	ZINC1853550	-7.2
				ZINC1087483	-7	ZINC35930738	-7.2
				ZINC1615742	-7	ZINC900708	-7.2
				ZINC5328058	-7	ZINC1530689	-7.2
						ZINC1689786	-7.1
						ZINC1670146	-7.1
						ZINC1934	-7.1
						ZINC100071772	-7.1
						ZINC3861600	-7.1
						ZINC4009000	-7
						ZINC1641089	-7

## Data Availability

The datasets provided in this study can be found in an online repository (https://www.ncbi.nlm.nih.gov/geo/query/acc.cgi?acc=GSE76427https://www.ncbi.nlm.nih.gov/geo/query/acc.cgi?acc=GSE102079https://www.cancer.gov/about-nci/organization/ccg/research/structural-genomics/tcga).
